# Innovative Mechanism of Rural Finance: Risk Assessment Methods and Impact Factors of Agricultural Loans Based on Personal Emotion and Artificial Intelligence

**DOI:** 10.1155/2022/1126489

**Published:** 2022-05-21

**Authors:** Na Zhao, Fengge Yao

**Affiliations:** ^1^Harbin University of Commerce, Harbin 150028, China; ^2^Qiqihar University, Qiqihar 161006, China

## Abstract

Agricultural finance is in an embarrassing position in the current financial environment, especially during the process of COVID-19. Based on a small-scale peasant economy, it can no longer meet the rapidly rising demand of farmers for agricultural finance. Moreover, there has been a serious disconnection between the financial system of secondary and tertiary industries, and the quality of development needs to be improved urgently. The agricultural loan risk assessment has always been the main problem that we pay great attention to in the innovation of agricultural finance. Agricultural loans are an indispensable element in supporting agricultural development and promoting rural revitalization strategy. However, financial institutions have certain credit risks in reviewing and issuing agricultural loans. This article studies the speech emotion recognition of farmers in loan review to assess loan risk. As for emotional confusion caused by speech segmentation, a special method of data connection between Convolutional Neural Networks (CNNs) and Bidirectional Long Short-Term Memory (Bi-LSTM) Networks is designed, and a variable-length speech emotion recognition model including CNN and Bi-LSTM is designed. Experimental results show that the proposed algorithm can effectively improve the risk assessment of farmers in loan review.

## 1. Introduction

Rural economic development is not only the purpose of rural revitalization but also the foundation and key to rural revitalization [1]. Rural economic development is inseparable from rural financial support. Agriculture has even become the bottleneck of China's economic development, which directly affects the coordinated development of China's social economy [2, 3]. There are not only the problems of the rural operation system itself but also the decentralization of operation mode, the transfer and reduction of the rural labor force in the process of urban-rural integration, the low comparative efficiency of agricultural products, and even the disconnection between the rural financial service system and the actual rural operation [4]. Since the reform and opening-up, China's rural financial system has been in active reform and achieved remarkable results. However, rural financial institutions lack a real endogenous financial system based on social finance in the case of the division of urban and rural capital elements, which leads to the plight of China's rural finance.

China is in the critical period of transition from the traditional small-scale peasant economy to large-scale modern agriculture. New agricultural entities have developed rapidly, but traditional farmers still account for the majority of agricultural production and management, which will coexist for a long time [5]. Facing this situation, rural finance should not only focus on supporting the development of new agricultural operation subjects but also meet the financial needs of the development of traditional smallholders' production and operation. Moreover, both new agricultural operators and traditional smallholders are also faced with the following problems: lack of independent property, insufficient assets that can be used for security, and lack of family and personal credit [6, 7]. How to design a rural financial system that can meet the financial needs of agricultural operating subjects and meet the fund security of rural financial institutions through innovation is still the key to the reform of the rural financial system.

China has more than 500 million rural residents: this huge population base indicates a broad rural financial market. However, even in the declining market of inclusive finance in recent years, the financial gap between agriculture, rural areas, and farmers in China is still 3 trillion yuan, and farmers' financing difficulties are still a big obstacle to rural economic development [8]. In the increasingly fierce financial market competition, small- and medium-sized rural banks (such as rural commercial banks and village banks) as a force should avoid stock competition with large state-owned banks and joint-stock commercial banks, focus on the rural financial incremental market, and provide traditional credit services for rural residents facing formal financial exclusion [9, 10]. According to the data of the third national agricultural census, the number of smallholders in China accounts for more than 98% of the main agricultural operators and 70% of the total cultivated land [11]. Farmers are still the main agricultural operators in China, and there is a general lack of effective collateral. Credit loans are the prospects for loan development. However, the weakness of agricultural operations and the instability of household income make the loan default risk higher, which is also the main cause of financial exclusion [12]. Therefore, the key to credit development of small- and medium-sized rural banks is to realize credit risk assessment of rural household loans and improve the identification ability of risk customers.

After investigation, we conclude that the risks of farmers' loans can be summarized as follows. (1) Preloan investigation risk: on the one hand, the risks are caused by the defect of farmers' own conditions; on the other hand, there is the game risk of information asymmetry between borrowers and banks. (2) Risk in farmers' loan: there are more risks in mortgage management. (3) Risk of postloan management of farmers' loans: postloan management is one of the key links to controlling loan risk. (4) Risks arising from the immaturity of the rural financial market: at present, the development of the rural financial market is not mature, mainly manifested by regional differences.

Over the past few decades, loan risk assessment has become an important basis for commercial banks to make reasonable financing decisions, reduce financing risks, and improve credit profits. Loan risk assessment methods include expert analysis, statistical analysis, and artificial intelligence (AI) [13, 14]. Studies have shown that AI has achieved better performance than statistical models in some loan risk assessment problems. Unlike statistical models, AI does not require assumptions about the distribution of variables and can derive knowledge directly from training datasets. In loan risk assessment, especially when the loan risk assessment problem is nonlinear pattern classification, the performance of AI is often better than the model based on statistical analysis. Given the above, we can conclude that the risk of farmers' loans is affected by many factors, and how to control the risk to the minimum has become the key to a point. It is urgent to introduce AI to analyze the risk assessment methods and impact factors of agricultural loans. In addition, when the bank-end reviews the loan matters, farmers' emotions can be recognized through voice recognition so as to make a more accurate risk assessment of farmers' loans.

The main contribution of this article is that a variable-length speech emotion recognition model, including Convolutional Neural Networks (CNNs) and Bidirectional Long Short-Term Memory (Bi-LSTM) Networks, is constructed.

## 2. Related Works

As the risk problem of commercial banks becomes more and more prominent, many scholars begin to pay attention to the study of loan risk assessment, and the main factors affecting loan risk become the focus of research. In [15], the authors put forward an optimal decision-making model for farmer credit based on a common risk guarantee fund and its application and constructed a nonlinear optimization model based on a risk compensation fund. In [16], the author combined the fuzzy comprehensive model with the fuzzy control model to construct the model and index system of credit risk characteristics of farmers in Yanliang, Shaanxi Province. In [17], the authors studied more than 1000 production and operation data samples of new agricultural subjects in three provinces of China and constructed an XGBoost model for empirical analysis. In [18], the authors proposed a credit risk approach that minimized the relatively high loss given default of highly rated loans as a risk rating grab criterion. In [19], the authors used delinquency of agricultural loans to approximate financial pressures and used logistic regression and several machine learning methods to predict financial pressures. In [20], the authors presented a credit risk assessment model to classify the credit rating of the borrowers of “three rurals.”

In this article, farmers' real-time emotions are analyzed by recognizing their speech emotions during loan reviews. Perceived emotions can be identified by changes in speech. For example, when people communicate with each other on the phone, they cannot see each other or sense their physical changes, such as blushing, while they can recognize the corresponding emotions of each other. Since emotions are related to many things, and speech is the easiest way for people to express emotions, it is of great significance to recognize the emotions of speakers through speech. In [21], the authors proposed a Focal Loss-based Convolutional Recurrent Neural Networks (FL-CRNN) deep learning model with variable input length for speech emotion recognition. In [22], the authors proposed an Automatic Encoder with Emotion Embedding (AEEE) to extract deep emotional features. In [23], Ozseven proposed a Statistical Feature Selection method based on the change of emotion on acoustic features (SFS-AF). In [24], Sun proposed an emotion recognition algorithm that did not rely on any speech acoustic features and combined the speaker's gender information. In [25], the authors proposed an emotion category-based feature weight method to find the significance of each feature under different emotions and take it as a priori knowledge.

## 3. Proposed Methodology

### 3.1. Variable-Length Speech Emotion Recognition Model Based on CNN and Bi-LSTM

In this section, a speech emotion recognition model with variable-length input based on CNN and Bi-LSTM is proposed, and a connection method between CNN and Bi-LSTM is designed. This model can accept speech input of different lengths without adjusting the model structural parameters. Thus, the whole sentence speech can be input into the model, and the emotion confusion caused by segmentation can be solved by feature extraction of the whole speech directly. Therefore, agricultural loan risk can be assessed by recognizing the speech of farmers in loan reviews.  Figure 1 shows the flowchart of the variable-length input emotion recognition algorithm based on CNN and LSTM.

Generally, the size of input data in neural network models is fixed, but the length of each speech sentence of farmers in agricultural loan review is basically different. Then, how to design an emotion recognition model so that it can receive variable-length input becomes a key problem. CNN is one of the most commonly used networks in deep learning classification tasks, whose characteristics of weight sharing and local connection greatly reduce the number of parameters. In the field of image recognition, CNN is usually used to process image input of the same size, and images of different sizes will be processed into the same size.

In fact, the reason why the size of CNN input needs to be fixed is that CNN usually connects the fully connected layer after using it. The input of the fully connected layer is a one-dimensional vector requiring a fixed length. CNN only performs two-dimensional convolution operations, and different input sizes will not affect the movement and convolution operation of the convolutional kernel. Output feature maps of different sizes can be obtained with different input sizes after convolution. Thus, when we design the speech emotional recognition model in agricultural loan review, feature extraction of CNN can proceed even if the input spectrogram size is different.

In the speech emotional recognition model in agricultural loan review, we introduce LSTM and design a data connection method that connects the CNN and LSTM after convolution. Bi-LSTM is adopted in this model. Compared with LSTM, Bi-LSTM overcomes the disadvantage that LSTM can only obtain updated information from the point before the current time point but cannot obtain information from the point after the current time point. Bi-LSTM can take into account both the information before the current time point and the information after the current time point. This is very important in the agricultural loan review; when farmers are asked questions about loans, there are maybe some conflicts with and in the dialogue. In the model, the dimension of Bi-LSTM's hidden layer state is set to 100, and the stack number of Bi-LSTM is two layers.

For Bi-LSTM, any output vector of Bi-LSTM contains information of all time points before this time point and information of all time points after this time point. The former is provided by the forward LSTM, and the latter is provided by the reverse LSTM. Therefore, each output vector contains relevant information on all time points. In this article, the output of the first neuron of LSTM and the output of the last neuron are combined as the output vector, which is connected to the fully connected layer to construct the global feature relationship. Finally, the classification results are output through the Softmax layer.

### 3.2. CNN + Bi-LSTM Connection Method

Bi-LSTM network cannot only meet the requirement of time sequence feature extraction but also meet the requirement of variable-length input. Apparently, the length of speech of farmers in loan review is not consistent. The design idea of variable-length input is similar to the coding part of the sequence to sequence process in Natural Language Processing (NLP) [26]. In NLP, different sentences will have different numbers of words, each word will be coded as a word vector, and then the word vectors of different sentences will be entered into the LSTM unit in sequence without any input problems caused by the irregular length.

Referring to this idea, the horizontal axis of the spectrogram is the frame number, which corresponds to the speech time length, while the longitudinal axis of the spectrogram corresponds to the frequency resolution of the speech. Its size is fixed and it is fixed to 256 in the experiment.

The spectrogram outputs the multichannel three-dimensional feature map after multilayer convolution and combines the longitudinal axis and channel axis of the three-dimensional feature map into a one-dimensional vector, while the horizontal axis corresponds to a one-dimensional vector per unit. These one-dimensional vectors have the same and fixed size, meeting the requirement of fixed input vector size for subsequent LSTM units. Then we get several eigenvectors and input them into the LSTM unit in turn according to the horizontal axis of the feature map. Then we can further extract the advanced features from CNN by utilizing the time information capturing capability of LSTM.

For example, we have a 256^*∗*^200^*∗*^1 size spectrogram and a 5^*∗*^4^*∗*^4 feature map after CNN processing. Then we merge the first dimension and the third dimension to get a set of two-dimensional vectors with a size o 20^*∗*^6, and the size of each one-dimensional eigenvector is 20. We input each eigenvector into LSTM in the order of the second dimension. A total of four LSTM units are required and the output results are finally obtained.

The design of this article not only solves the problem of variable-length input but also constructs the time sequence relationship between the front and back of speech after Bi-LSTM processing. The output of the network includes the time sequence features of speech. Therefore, the results are more suitable for speech feature extraction and analysis.

## 4. Experiment and Results Analysis

### 4.1. Datasets

The experiment uses the AISHELL-1 Mandarin corpus, which is a Mandarin speech dataset with a sampling rate of 16000 Hz [27]. Among them, the training set, verification set, and test set contain 120098, 14326, and 7176 standard corpora, respectively, with a total data duration of about 178 h, and there is no overlap among the corpus of the training set, verification set, and test set. The output emotions are classified into four categories: anger, happiness, neutral, and sadness.

For the final model test, dialogues of datasets will be randomly selected in this article. In total, 80% of dialogues of the corpus are randomly selected as the training set and the remaining 20% as the test set. In this way, the identity of the speaker cannot be accurately known even in the prediction process of the final model, ensuring the universality of the final prediction model in agricultural loan review. The PyTorch framework is used for model construction in the experiment. The cross-entropy loss function is used in the model training process in the experiment, and the stochastic gradient descent method is adopted for optimization. The learning rate of training is 0.001, and the number of batch training is 8.

### 4.2. Parameters Setting

The overall process is shown in Figure 2. The CNN part of the model consists of three convolution layers. Farmers' speech data in agricultural loan review is sent to Bi-LSTM after being connected after CNN output. The hidden layer state dimension of Bi-LSTM is set to 50, and the stack number of Bi-LSTM is set to 2. After output from Bi-LSTM, the farmers' speech data in the agricultural loan review enter the fully connected layer to construct the global feature relationship and finally output the classification results through the Softmax layer. The specific steps are defined as follows.

The input of the model's spectrogram is the whole sentence spectrogram with a size of 1^*∗*^156^*∗*^*N*, where *N* is the number of frames after the speech of different lengths is converted into the spectrogram.

#### 4.2.1. CNN Part

The first layer is the convolutional layer. The step size is set to 2 and the padding is set to 0. It is composed of 64 kernels with a size of 12^*∗*^15. The maximum pooling method is used. The size of the pooling layer is 2^*∗*^2 and the step size is 2. After the convolutional pooling of the first layer, the feature map size is 64^*∗*^64^*∗*^*N*_1_, and *N*_1_ is the spectrogram with a number of frames *N*, that is, the size of the horizontal axis of the feature map after the convolutional layer processing of the spectrogram with the horizontal axis *N*, and the corner marker represents the serial number of the convolutional layer. The second layer is the convolutional layer. The step size is set to 2, the padding is set to 0, and 128 kernels with a size of 15^*∗*^18 are used. The maximum pooling method is used. The size of the pooling layer is 2^*∗*^2, the step size is 2, and the padding is 0. The size of the feature map obtained after the second convolutional pooling process is 128^*∗*^12^*∗*^*N*_2_. The third convolutional layer only has convolution operation with 2 steps and 0 paddings, which is composed of 128 kernels with size 4^*∗*^4. The size of the feature map after convolution is 128^*∗*^4^*∗*^*N*_3_.

#### 4.2.2. Data Connection Part

The final output size of CNN is 128^*∗*^4^*∗*^*N*_3_, and the output is 512^*∗*^*N*_3_ after processing of data connection.

#### 4.2.3. Bi-LSTM Part

The obtained feature data with a size of 512^*∗*^*N*_3_ is regarded as *N*_3_ one-dimensional eigenvectors with a size of 512. Each eigenvector is sequentially input into Bi-LSTM network along the *N*_3_ dimension, and the output of the first neuron and the output of the last neuron are combined as the output vector.

#### 4.2.4. Fully Connected Layer

The final output of Bi-LSTM is a one-dimensional vector of size 200^*∗*^1, which is input into the fully connected layer with an output size of 4^*∗*^1. Then, the value is normalized to the range of [0,1] by the Softmax function to output the classification recognition probability.

### 4.3. Evaluation Method

The experiment uses two general metrics and a confusion matrix to evaluate the performance of the model.

(1) Weighted accuracy (WA), which is defined as equation (1), is the percentage of correct samples of all sentences in the test set.
(2) Unweighted accuracy (UA), which is defined as equation (2), is each type of emotional accuracy calculated separately, and then the average accuracy is obtained.
  (1) $$\begin{array}{c} WA=\frac{\sum_{k-1}^{n}TP_{k}}{\sum_{k-1}^{n}\left(TP_{k}+FN_{k}\right)}, \end{array}$$
  (2) $$\begin{array}{c} UA=\frac{1}{n}\sum_{k-1}^{n}\frac{TP_{k}}{TP_{k}+FN_{k}}, \end{array}$$
where *n* is the number of emotion categories, *TP*_*k*_ represents the number of correctly predicted *k* th samples, and *FN*_*k*_ represents the number of incorrectly predicted *k* th samples.

### 4.4. Spectrogram Extraction

The spectrogram is extracted by librosa tool library in Python to extract frame-level spectral features from speech signals of farmers' agricultural loan review. Each frame is divided into 50 ms by hamming window, and there is 8 ms overlap between frames. Afterwards, a discrete Fourier transform of 1024 length is applied to each frame, and its power spectrum is obtained to obtain multiple short-time spectrums. By sorting the spectrum in chronological order, the final spectrogram is obtained. However, for the speech emotion recognition model with variable-length input, we change the processing method of the spectrogram. The purpose of our improvement is to realize the input of the whole sentence and avoid the confusion of neutral and nonneutral emotions caused by segmentation. Therefore, the following different processing methods of the spectrogram are adopted in designing the input of the spectrogram:

1. *No Padding*. The spectrogram of each speech is directly input into the model. However, due to the different length of each speech, the length of each spectrogram is different, so the training process of the model can only be conducted once.
2. *Batch Padding*. To avoid the problem of low efficiency of single training, spectrograms with similar lengths are placed in the same training batch, and these spectrograms are filled to the same length by zeroing operation, with 100 frames as the unit and 100 frames as the difference, so as to facilitate the training of the model.
3. *Maximum Length Padding*. The purpose is to compare the recognition model of fixed-length input after speech segmentation. The spectrogram of the whole sentence is filled to the maximum length of all spectrograms, which in this experiment is filled to 1300 frames.

### 4.5. Experimental Results and Analysis

Experiments are performed on the fixed-length farmers' speech in agricultural loan review emotion recognition model based on CNN and the variable-length speech emotion recognition model based on CNN + Bi-LSTM, and the recognition accuracy is tested. A total of 300 cycles of training were performed in the experiment, and the model achieved the optimal recognition effect at 164 times; then, we saved the model. WA and UA are used to represent the overall emotion recognition performance of the model. The recognition accuracy of each model structure is shown in Tables 1and 2.

The experimental results show that the accuracy of fixed-length farmers' speech in the agricultural loan review emotion recognition model is 80.14% for WA and 76.87% for UA. The accuracy of the variable-length farmers' speech in the agricultural loan review emotion recognition model is 85.61% and 80.73% for WA and UA, respectively. Compared with the fixed-length farmers' speech in the agricultural loan review emotion recognition model, the recognition rate increases by 6.83% and 5.02%, respectively, indicating that the improvement of the input into the spectrogram of the whole sentence speech has a good effect on the improvement of recognition rate.

To make a full comparison of the effects, the old spectrogram image segments with fixed length after segmentation are used as input to the new CNN + Bi-LSTM-based model. The recognition rate increased by 4.62% compared with the old CNN-based model. This shows that Bi-LSTM improves the accuracy of the model compared with the model using only CNN. These results indicate that using LSTM to retain the sequential characteristic of speech signal can improve the effect of farmers' speech in agricultural loan review emotion recognition. In the training experiment results of the variable-length farmers' speech in the agricultural loan review emotion recognition model, the accuracy of the training set without padding input is maintained at 57.44% after 41 rounds of cycle training. At this time, WA and UA of the test set are 61.55% and 45.00%, respectively. After 118 cycles of batch padding input, the training set achieves an accuracy of 93.46%, while the test set has the best recognition accuracy, which is 85.61% for WA and 80.73% for UA. When the maximum length padding input is 152 epochs, the accuracy of the training set reaches 96.77%, and the test set has the best recognition accuracy, which is 84.99% for WA and 79.43% for UA.

As for the problem that the accuracy of the training set without padding input stays at 57.44%, we put forward two possibilities: one is that the training model may fall into local minimum due to the small step of gradient descent; second, due to insufficient model complexity, the underfitting occurs. Therefore, we test for this. Firstly, starting from solving the local minimum problem, after trying to increase the learning rate to try different values, it is found that the problem has not been improved. When the CNN model is directly replaced by the classical complex neural network ResNet-50, the problem is solved. According to the above test results, the reason for the low accuracy of the training set without padding input is the insufficient complexity of the model, and the problem of underfitting occurs. The biggest difference between batch input and maximum length input and no input is batch training. Batch training makes the model fitting effect better and overcomes the underfitting problem to some extent, achieving good results. According to the experimental results, WA input of batch padding is 0.34% lower than that of maximum length padding, and UA is 2.21% higher than that of maximum length padding. We analyze that the WA of batch padding input is low because the input length of each batch is different, which makes it more difficult for the model to acquire various emotional features in speech. However, the UA of the maximum length padding is low because there are too many zero-padding operations in the maximum length padding, and the existence of 0 value in the process of maximum pooling has an impact. Nevertheless, the recognition accuracy of the two models is significantly improved compared with that of the fixed-length farmers' speech in the agricultural loan review emotion recognition model.

To further achieve the purpose of this paper and analyze the improvement effect of recognition accuracy brought by variable-length input, we present the confusion matrix of the fixed-length agricultural loan review emotion recognition model based on CNN in Figure 3 and the confusion matrix of the maximum length padding variable-length agricultural loan review emotion recognition model in Figure 4. In Figure 5, the confusion matrix of batch padding input in the variable-length farmers' speech in the agricultural loan review emotion recognition model is given.

Based on the confusion matrix results, anger has the highest recognition rate in the emotion classification of fixed-length farmers' speech in the agricultural loan review emotion recognition model, while happiness and neutral emotions have lower recognition rates. This may be due to the confusion between neutral and nonneutral emotions. Not all parts of the nonneutral sentence contain nonneutral emotions. During the process of fixed-length farmers' speech in agricultural loan review emotion recognition, these neutral clips are segmented and labeled with nonneutral emotions, which makes the model unable to distinguish the characteristics between labels very well. Compared with the fixed-length model, the neutral emotion recognition rate of the variable-length model is improved, and the whole sentence is input into the network, which reduces the confusion of neutral emotions and other emotions caused by segmentation. The accuracy of happiness has also been improved, indicating that happy-related sentences contain neutral speech segments that are labeled as happiness when using input model segmentation with fixed-length farmers' speech in agricultural loan review; thus, the model cannot learn happiness characteristics well. Recognition rates for anger and sadness are reduced, possibly due to the fact that model parameters with constant input do not achieve the best results.

From the above experimental results, we can conclude that the neutral emotion confusion caused by sentence segmentation is improved after the input of fixed-length segmentation changes to that of the whole sentence. However, the model proposed in this article is not the optimal state. When the input changes to the whole sentence input, the number of speech emotional features increases, while some features have a low value for emotion recognition, which requires the model to be more optimized. Therefore, updating the model for variable-length input is helpful to further improve the recognition accuracy.

In addition, for the risk assessment of agricultural loans, we use speech recognition to classify the voice of farmers in loan review and then judge whether the farmers conceal the loan-related matters or not. Figures 6and 7 are the accuracy and classification time of the CNN + Bi-LSTM algorithm and the other three baselines, respectively. As can be seen from Figure 6, the accuracy of the algorithm proposed in this article has always been the highest, all above 90%, which is very important in loan evaluation. Higher accuracy is accompanied by the accuracy of speech recognition, which is helpful for farmers' loan review. On the contrary, the performance of the three baselines is not conducive to the classification of farmers' speech recognition emotion during loan review.  Figure 7 shows the comparison of classification time. The classification time of the algorithm proposed in this article has always been the lowest. In risk assessment of loan, besides the accuracy of speech emotion recognition, the classification time is also very important. Speech can well reflect the change of emotion, but the instantaneous change of tone may lead to the fluctuation of emotion, which is important for loan evaluation to be detected through speech emotion recognition.

## 5. Conclusions

This article studies the innovative mechanism of rural finance and constructs a risk assessment model of agricultural loans based on farmers' speech in agricultural loan review emotion recognition in loan review for the confusion of neutral emotion and nonneutral emotion caused by speech segmentation of fixed-length speech emotion recognition algorithm. In this article, a variable-length input speech emotion recognition model is proposed, and a connection method between CNN and Bi-LSTM is designed. Without changing the structural parameters of the model, the whole farmers' speech in agricultural loan review of different length can be sent into the model as input, which overcomes the problem of fixed input length of the neural network. The experimental results show that the variable-length input method can effectively solve the confusion problem of neutral emotion and three kinds of nonneutral emotion in agricultural loan review, which greatly improves the recognition accuracy of the model.

With the further deepening of the research, the following aspects can be improved in the follow-up research work: (i) this paper focuses on the research of the discrete emotional model, while the discrete emotional model simplifies the continuous state of emotion. In the follow-up work, it is necessary to increase the research on the continuous emotional description model and construct a continuous emotional change tracking curve. (ii) For the application of farmers' speech in agricultural loan review emotion recognition, the ability of speech emotion recognition to cross-database and cross-platform generalization should be improved to realize real-time detection of individual emotional changes. (iii) In the study of agricultural loan risk assessment, we should perfect and unify the farmers' credit assessment system, establish a complete database to form dynamic tracking, and improve the accuracy and applicability of loan risk assessment. (iv) The research topic of this article is the risk assessment of the farmers in loan review. The relevant speech emotion recognition model constructed in this article can be further applied to the customer loss of banks, credit card fraud recognition, and other fields to verify the applicability of the model and expand the corresponding research field.

## Figures and Tables

**Figure 1:** Variable-length input speech emotion recognition model.

**Figure 2:** Flowchart of CNN + Bi-LSTM-based variable-length input speech emotion recognition.

**Figure 3:** CNN-based confusion matrix of fixed-length emotion recognition model.

**Figure 4:** CNN + Bi-LSTM-based confusion matrix of maximum length padding variable-length emotion recognition model.

**Figure 5:** CNN + Bi-LSTM-based confusion matrix of batch padding variable-length emotion recognition model.

**Figure 6:** Accuracy of farmers' speech emotion recognition in loan review.

**Figure 7:** Classification time of farmers' speech emotion recognition in loan review.

**Table 1:** Accuracy of fixed-length farmers' speech in agricultural loan review emotion recognition model based on CNN.

Model	WA (%)	UA (%)
Three convolutional layers	77.92	74.10
Five convolutional layers	80.14	76.87
ResNet-18 layers	78.19	71.36

**Table 2:** Accuracy of variable-length farmers' speech in agricultural loan review emotion recognition model based on CNN + Bi-LSTM.

Model	Spectrogram input form	WA (%)	UA (%)
Three convolutional layers + Bi-LSTM	Fixed-length input	84.26	77.01
Three convolutional layers + Bi-LSTM	No padding input	61.55	45.00
Three convolutional layers + Bi-LSTM	Batch padding	85.61	80.73
Three convolutional layers + Bi-LSTM	Maximum length padding	84.99	79.43

## Data Availability

All data used to support the findings of the study are included within this article.
